# Diagnostic and Therapeutic Roles of Extracellular Vesicles in Aging-Related Diseases

**DOI:** 10.1155/2022/6742792

**Published:** 2022-08-08

**Authors:** Zixuan Sun, Xiaomei Hou, Jiaxin Zhang, Jiali Li, Peipei Wu, Lirong Yan, Hui Qian

**Affiliations:** ^1^Department of Gerontology, Affiliated Hospital of Jiangsu University, Zhenjiang 212001, China; ^2^Key Laboratory of Laboratory Medicine of Jiangsu Province, School of Medicine, Jiangsu University, Zhenjiang 212013, China

## Abstract

Aging shows a decline in overall physical function, and cellular senescence is the powerful catalyst leading to aging. Considering that aging will be accompanied with the emergence of various aging-related diseases, research on new antiaging drugs is still valuable. Extracellular vesicles (EVs), as tools for intercellular communication, are important components of the senescence-associated secretory phenotype (SASP), and they can play pathological roles in the process of cellular senescence. In addition, EVs are similar to their original cells in functions. Therefore, EVs derived from pathological tissues or body fluids may be closely related to the progression of diseases and become potential biomarkers, while those from healthy cells may have therapeutic effects. Moreover, EVs are satisfactory drug carriers. At present, numerous studies have supported the idea that engineered EVs could improve drug targeting ability and utilization efficiency. Here, we summarize the characteristics of EVs and cellular senescence and focus on the diagnostic and therapeutic potential of EVs in various aging-related diseases, including Alzheimer disease, osteoporosis, cardiovascular disease, diabetes mellitus and its complications, and skin aging.

## 1. Introduction

Extending the human lifespan is a major goal of medical research, and aging seems to be a stumbling block to human longevity. It is a multifactorial biological process accompanied with the accumulation of senescent cells and the decline of body function [1, 2]. The physiological role of cellular senescence depends on the recruitment of immunocytes by senescent cell-secreted senescence-associated secretory phenotype (SASP) factors. However, after exerting their beneficial effects, the senescent cells cannot be completely cleared by the immune system [3]. Sustained secretion of SASP factors could lead to chronic inflammation, which is an essential contributor to aging-related diseases [4]. Senescent cells are mainly characterized by changes in nuclear genes, mitochondrial and lysosomal system dysfunction, and increased SASP factor secretion [5, 6]. Numerous studies have confirmed the key roles of extracellular vesicles (EVs) in DNA damage repair, inflammatory regulation, and epigenetic alterations, showing their great medical value in aging-related diseases.

EVs are diverse nanoscale membrane vesicles secreted by most cell types [7]. Based on their biogenesis, size, and biophysical properties, they can be classified into apoptotic bodies, exosomes, and microvesicles (MVs) [8]. In the process of the synthesis and secretion of EVs, signaling molecules such as DNA, RNA, functional proteins, and lipids can be selectively encapsulated, indicating the sharing of biological information among cells [9]. EVs are important components of SASP factors, and their information transmission function plays a vital role in cellular senescence [5, 10]. Particularly, senescent cells can promote the senescence of surrounding bystander cells by secreting SASP factors [11]. In addition, senescence manifests a decline or even loss of stem cell proliferative capacity, so stem-cell therapy has also emerged. However, due to the uncontrollable differentiation of stem cells, it may have carcinogenic and teratogenic effects, and the surgical cost is high. Compared with cell therapy, EVs are similar to their parent cells in functions, and they have the advantages of low carcinogenicity and no blockage of blood vessels, which make EVs become promising antiaging agents [12]. In this review, we summarize the roles of different sources of EVs as biomarkers and treatments of various aging-related diseases, and the current knowledge around the challenges and prospects of EVs are also discussed.

## 2. EVs as Biological Tools for Cell Communication

The effectiveness of EVs mainly depends on which cargoes they carry. In fact, the current researches on the pathogenic and therapeutic effects of EVs are mainly based on the belief that EVs can be used as tools for intercellular information transmission. As an important member of EVs, the exosome also plays a major role in cell communication. At present, it is believed that the biogenesis of exosomes originates from the endosomal pathway [13] (Figure 1). Endocytic vesicles form and fuse on the plasma membrane to form early endosomes. Next, early endosomes sink again and mature to form late endosomes. These late endosomes are also known as multivesicular bodies (MVBs) [14], which contain intraluminal vesicles (ILVs) formed through endosomal sorting complex required for transport- (ESCRT-) dependent and ESCRT-independent pathways [15–17]. The formation of ILVs is accompanied by cargo loading, which is crucial for cell communication. After vesicular accumulation, some MVBs are degraded in lysosomes, and the other MVBs release ILVs out of cells by fusing with the plasma membrane. These ILVs are the precursors of exosomes [18]. The uptake of exosomes by recipient cells is another important step in cell communication (Figure 1). Exosomal cargoes are internalized into recipient cells through a variety of mechanisms: (i) receptor-mediated phagocytosis of special cells, (ii) megapinocytosis of plasma membrane invagination, and (iii) direct fusion with the plasma membrane [19]. The cargoes of exosomes could change the state of recipient cells or make them obtain new abilities, which reflects the medical value of exosomes [20].

## 3. Stimuli and Characteristics of Cellular Senescence

The accumulation of senescent cells *in vivo* is an essential mechanism of aging [21], and it is also the culprit of aging-related diseases. Although cell senescence has certain physiological effects [2, 22], excessive senescent cell accumulation can create a proinflammatory environment conducive to the occurrence and development of aging-related diseases [23] (Figure 2).

Although cellular senescence is a complicated process [6, 24], it can be summarized into two basic events: the change of nuclear genes and the transformation of mitochondria [5]. The changes of nuclear genes include DNA damage, telomere shortening, and epigenetic change [25]. The mitochondrion is a multifaceted regulator of aging [26]. The loss of mitochondrial DNA integrity and destruction of mitochondrial metabolism are regarded as evolutionarily conserved senescent mechanisms [27]. In fact, mitochondrial dysfunction is associated with low NAD^+^/NADH ratios [28] and high level of SASP factors and reactive oxygen species (ROS) [29, 30]. Because of the complexity of the cellular senescence mechanism, the characteristic of senescent cells shows complex dynamics and heterogeneity. Therefore, the identification of senescent cells involves many aspects [21] (Figure 2). There is still no gold standard for identifying senescent cells [31], and the combination of multiple aging phenotypes to identify senescent cells is still the best choice at present [32]. In order to further explore the diagnosis and treatment of aging-related diseases, it is very important to clarify the stimuli and characteristics of cellular senescence.

## 4. EVs in Aging-Related Diseases

Aging is characterized by the disorder of various biological functions, which leads to an increased risk of osteoporosis, diabetes mellitus (DM), cardiovascular diseases (CVDs), Alzheimer disease (AD), and other chronic diseases [33]. Increasing researches have demonstrated that EVs can serve as potential biomarkers and therapeutic reagents in aging-related diseases. Here, we introduce the most studied aging-related diseases in the field of EVs (Figure 3).

### 4.1. Roles of EVs in AD

Around the world, AD is a leading cause of disability in people over 65 years old [34]. Two main histopathological features of AD are (i) senile plaques formed by increased deposition of the amyloid beta (A*β*) peptide and (ii) intracellular neurofibrillary tangle (NFT) caused by tau hyperphosphorylation [35]. Aging is a major risk factor for AD [36], and cellular senescence is one of the hallmarks of aging, which increases susceptibility to AD. Enrichment of senescent astrocytes, microglia, and neurons, as well as the expression of senescence-associated *β*-galactosidase (SA *β*-Gal), were observed in the brain tissue of AD patients [37]. Senescent astrocytes and microglia could promote tau hyperphosphorylation [38]. It is suggested that clearing senescent nerve cells might be helpful to inhibit the occurrence of AD. In addition, AD has a longer preclinical phase [39], and the onset of clinical symptoms can be alleviated if treatment is available in this period [34]. Therefore, biomarkers for the early diagnosis of AD is urgently needed.

#### 4.1.1. EVs as Low-Invasive Markers for Early Diagnosis of AD

At present, the combined detection of A*β*42, total tau (t-tau), and phosphorylated Thr181 tau (p181-tau) in the cerebrospinal fluid is the gold standard for the diagnosis of AD [40]. However, this method requires invasive lumbar puncture to obtain cerebrospinal fluid, limiting its clinical application. Positron emission tomography (PET) has been proven to have high accuracy in AD diagnosis *in vivo*, but it is not available in most medical settings [41]. Therefore, the detection of blood-based biomolecules that are less invasive and easy to implement have become alternative methods for AD diagnosis.

Recently, EVs isolated from peripheral blood have aroused the interest of researchers. Longobardi et al. [42] found that patients with different types of dementia have differences in the size and number of blood-derived EVs, indicating that their physical characteristics might be promising markers for dementia. In addition, EVs contain the A*β* peptide and tau that play important roles in the occurrence of AD. This presents their great potential in the diagnosis of AD. Delgado-Peraza et al. [43] reported that in AD mouse models, plasma neuronal EVs (NEVs) carry higher levels of t-tau, p181-tau, and A*β*42, and those astrocytic EVs (AEVs) carry higher levels of complement proteins. The levels of these markers in plasma NEVs and AEVs are correlated with their levels in brain tissue, thus supporting the use of plasma EV biomarkers for detecting brain pathology. Similarly, changes in other forms of A*β* peptide and tau have also been found in AD patients [39, 41, 44]. Besides, there are several other promising biomarkers based on EVs for AD diagnosis, such as matrix metalloproteinase 9 (MMP-9), growth-associated protein 43 (GAP43), neurogranin, synaptosome-associated protein 25 (SNAP25), and synaptophysin 1 [34, 41]. Notably, in addition to using EVs alone, some researchers have combined olfactory functions with A*β*1-42 and Sniffin' Sticks (SS-16) to more accurately predict the transition from mild cognitive impairment to AD dementia [45] (Table 1).

#### 4.1.2. Roles of EVs from Different Sources in AD Treatment

Due to the heterogeneity of EVs, those EVs from healthy cells can act therapeutically on AD. Li et al. [46] injected neural stem cell-derived EVs (NSC-EVs) into the lateral ventricle of AD mice and found that the mouse inflammatory response was reduced and cognitive impairment was rescued. Similarly, Apodaca et al. [47] injected NSC-EVs intravenously into 5xFAD mice. And EV treatment reversed the cognitive impairment of AD mice by reducing A*β* plaques, inhibiting microglia activation, and promoting synaptophysin recovery in the brain. Several potential therapeutic EV cargoes were identified by using TaqMan Advanced miRNA Assays, including miR-125b-5p, miR-124-3p, and miR-125a-5p, thereby providing candidate miRNAs for follow-up studies. In addition, EVs derived from mesenchymal stromal cells (MSC-EVs) have shown good therapeutic effects on AD [48–50]. Besides, a recent study found that ultrasound could increase the release of exosomes derived from human astrocytes (HAs) by nearly five times, and these exosomes demonstrated excellent therapeutic effects, suggesting that applying physical methods may help solve the problem of low EV yields [51].

Because of EVs' advantages of homing ability, good biocompatibility, and blood-brain barrier penetration, they can serve as excellent drug carriers. By using plasma exosomes to load quercetin (Que), Qi et al. [52] found that Exo-Que could remarkably improve brain targeting and bioavailability of Que. Compared with free Que, Exo-Que inhibited tau phosphorylation and the formation of NFT, which could better alleviate the symptoms of AD, indicating that Exo-Que has better potential for the treatment of AD (Table 2). This represents the positive function of EVs in drug delivery, but the loading efficiency should also be considered.

### 4.2. Roles of EVs in Osteoporosis

Osteoporosis can lead to bone fragility and an increased risk of fractures [62, 63]. Osteoporotic fractures are most commonly found in the spine, hip, or wrist [64], and it is a major cause of global health expenditures. As a unique tissue form, the bone can heal without fibrous scars. But healing disorders associated with osteoporotic fractures, especially nonunion, will prolong treatment time and increase the socioeconomic burden [65]. The risk of fracture in patients with osteoporosis is mainly due to the increased bone resorption caused by the increased activity of osteoclasts. Moreover, that osteoblasts cannot make up for this bone loss in time will result in serious delays of bone reconstruction [66].

#### 4.2.1. Pathological Roles of EVs in Osteoporosis

At present, the researches on the pathological mechanisms of osteoporosis mainly focus on the functional imbalance between osteoblasts and osteoclasts, as well as the imbalance between osteogenic differentiation and adipogenic differentiation of bone marrow MSCs (BMSCs) [67, 68]. DNA damage, apoptosis, and cellular senescence induced by oxidative stress are important reasons for the imbalance of the bone tissue environment [69]. As essential participants in the aging process, EVs make a difference in the imbalance of bone homeostasis and the occurrence and development of osteoporosis. Additionally, the communication function of EVs determines their crosstalk abilities between cells and tissues in the pathological process of osteoporosis. Crosstalk between the bone and muscle is a new research direction. Some researchers have reported that muscle-derived EVs carrying miR-34a could induce BMSC aging by reducing sirtuin 1 (SIRT1) expression in BMSCs, thus decreasing bone mass [70]. Angiogenesis, a key factor in bone reconstruction, can be regulated by the bone itself. Senescence osteoblast-derived exosomes could upregulate miR-139-5p expression in vascular endothelial cells. miR-139-5p acts on the target gene TBX1, which could increase aging and apoptosis and reduce the proliferation and migration of vascular endothelial cells, thus affecting the process of osteoporosis [71]. Therefore, blocking the transmission of harmful EV has become a potential therapeutic target for osteoporosis.

#### 4.2.2. Calcification Paradox in Aging

The great significance of the calcification paradox in aging deserves attention. The calcification paradox means that vascular calcification (VC) and osteoporosis are often accompanied in the elderly population. VC is an early pathological change in many CVDs [72], and it also promotes osteoporosis by damaging the blood and nutrient supply of cortical bone [73]. A recent study revealed the molecular mechanism of the calcification paradox: (i) miR-483-5p in the aged bone matrix-derived EV (AB-EV) targets BMSCs to promote their adipogenic differentiation rather than osteogenic differentiation, thus promoting osteoporosis, and (ii) miR-2861 in AB-EVs promotes the ossification of vascular smooth muscle cells, thus promoting vascular calcification [74]. Notably, young BMSC-EVs not only promote osteogenesis in bone but also inhibit phosphate-induced VC in the vascular system [75, 76]. This suggests that young BMSC-EVs can regulate mineral disorders, and we should also pay attention to the impact on other systems when studying the effect of EVs on one disease.

#### 4.2.3. Targeted Therapy of EVs from Different Sources in Osteoporosis

The treatment of osteoporosis depends on drugs, mainly antiresorptive agents, such as bisphosphonates, while the drugs approved by the FDA to restore bone loss are only parathyroid hormones (PTHs) [77, 78]. In addition to medication, physical therapy for osteoporosis, such as external mechanical load, can improve bone quality by promoting angiogenesis and driving BMSC recruitment and differentiation [79, 80]. The osteoporosis model used in a recent study is based on this principle. Specifically, this model suspended the hind legs of mice to eliminate mechanical load [81]. However, Xun et al. [78] found that this method was not effective at all ages. By contrast, fatigue load aggravated the microdamage of tibias in elderly osteoporotic rats, and the osteogenic differentiation ability of BMSCs was also decreased. In general, the therapeutic methods of osteoporosis still need to be expanded.

The therapeutic effect of EVs on osteoporosis is mainly reflected in promoting angiogenesis, inhibiting proliferation and differentiation of osteoclasts, and promoting the proliferation and osteogenic differentiation of BMSCs (Table 2). In addition to osteoblasts and osteoclasts, BMSCs are also key components in new bone formation. The adipogenic differentiation tendency of BMSCs is considered an essential cause of osteoporosis [82]. This is consistent with increased adipogenesis and decreased bone formation in osteoporosis [63]. Therefore, BMSC is the preferred therapeutic target for osteoporosis. Sonoda et al. [83] first demonstrated that systemic infusion of EVs derived from stem cells from human exfoliated decimal teeth could regulate telomerase activity, thereby improving the damaged function of BMSCs. Similarly, EVs derived from the mid-to-late stages of osteoblast differentiation could be helpful to restore the normal osteogenic differentiation level of BMSCs [84]. Although many studies have confirmed the therapeutic effect of EVs on osteoporosis, there is still a lack of optimal choice of the source of EVs. Good bone targeting is the guarantee for EVs to treat osteoporosis *in vivo*. Considering the homing ability of MSC-EVs, EVs from BMSCs are mostly selected in EV research on osteoporosis [63, 82, 85–87]. Although the bone-targeting ability of BMSC-derived exosomes (BMSC-Exos) is greatly improved compared with first-line osteoporosis drugs, such as bisphosphonates, their targeting ability may need further confirmation. EVs derived from vascular endothelial cells (ECs) and mid-to-late stages of osteoblast differentiation also exhibit innate bone-targeting potential [84, 88]. Notably, Lou et al. noted that although bone marrow stromal cell- (ST-) derived exosomes have a therapeutic effect *in vitro*, they failed to prevent postmenopausal osteoporosis induced by ovariectomy in the mouse model [77]. However, by binding BMSC-targeting aptamers to ST-derived exosomes, this complex could effectively accumulate in the bone marrow and showed a therapeutic effect *in vivo*. This suggests that engineering EVs to enhance their bone targeting is feasible. Similarly, Wang et al. linked alendronate to mouse MSC- (mMSC-) derived EVs by click chemistry, which not only improved bone targeting but also alleviated the side effects of alendronate [89]. While ensuring the efficacy, the availability of EV sources is another consideration. Human umbilical cord mesenchymal stromal cells (hucMSCs) [81], bovine milk [90], bovine colostrum [91], human amniotic fluid stem cells (hAFSCs) [92], and human umbilical cord blood (hUCB) [93] have unique source advantages. Since EVs derived from senescent cells carry aging information and have pathogenic potential, it is necessary to ensure that EVs come from young cells or body fluids [93]. In conclusion, the ideal source of EVs should have the characteristics of good bone targeting, easy availability, and coming from young individuals. Unfortunately, the study on the molecular mechanism of EVs in the treatment of osteoporosis is still very limited. This is undoubtedly a future research direction.

### 4.3. Roles of EVs in CVDs

Age is the primary risk factor for CVDs [104]. By 2030, 23.6 million people are expected to die annually from CVDs [105], which has aroused great attention to cardiovascular health all over the world. Recently, EVs have emerged as new players in the researches on pathology, diagnosis, and treatment of CVDs.

#### 4.3.1. Cardiovascular Aging

Vascular aging occurs before clinical diseases and can lead to serious CVDs [106, 107]. It mainly occurs in the inner and middle layers of the vascular wall [107]. Therefore, as the main cells of the blood vessel wall, ECs and vascular smooth muscle cells (VSMCs) play vital roles in vascular aging. During vascular aging, tube wall stiffness and compliance decrease. Women exhibit higher wall hardness than men [108]. The mechanism underlying this association may explain sexual differences in the incidence rate of CVD. In addition to blood vessels, the function of the heart decreases with age. Increases in heart mass and volume and a decreased maximum heart rate are the main characteristics of heart aging [108]. Notably, changes in the cardiomyocyte structure and function precede anatomical and functional changes in the heart [109]. Mitochondria are critical for heart aging, which is consistent with the mechanism of cellular senescence. Apart from affecting the energy transfer efficiency of cardiomyocytes [110], mitochondrial acetaldehyde dehydrogenase (ALDH2) can also influence cardiac aging by affecting autophagy [111]. Dysfunction associated with cardiovascular aging will lead to various CVDs.

#### 4.3.2. Hypertension

The main harm of hypertension is to damage cardiovascular and renal health [112]. Since the etiology of hypertension is still not clear, the current research on EVs in the treatment of hypertension is mainly aimed at the accompanying cardiovascular and renal injury. For example, plasma exosomes could regulate the structure and function of cardiovascular tissue and systemic blood pressure in hypertensive rats [94]. And exosomes secreted by cardiosphere cells could treat angiotensin II-induced hypertension-related myocardial hypertrophy and renal injury [95]. Vascular remodeling is a key event in the development of hypertension. Considering that ECs and VSMCs are essential in vascular remodeling, these two cells are important therapeutic targets for vascular injury induced by hypertension [113]. In addition, in view of the correlation between hypertension and aging, cellular senescence-related signal pathways and molecules deserve attention while studying the specific mechanism of EVs on hypertension. There is no doubt about the close relationship between MMPs and aging. In fact, MMPs can participate in skin aging [114], neurodegenerative diseases [115], and hypertension. By activating the SIRT1-AMPK*α*-eNOS pathway and downregulating MMPs, EVs from induced pluripotent stem cell- (iPSC-) derived MSCs could reduce aging-related vascular endothelial dysfunction and hypertension [96]. Besides, oxidative stress [116] and chronic inflammation [117], the risk factors of aging are also the targets of EVs in the treatment of hypertension. miR-155-5p in adventitia fibroblast-derived EVs under normal blood pressure could inhibit the proliferation and migration of VSMCs under hypertension by inhibiting oxidative stress, inflammation, and the expression of the angiotensin-converting enzyme [97, 98]. It should be noted that different hypertensive mouse models may reveal different results in the study of hypertension mechanisms and treatment, and the impact of this difference should be excluded as far as possible in practical research (Table 2).

The early diagnosis of aging-related diseases is of great significance for disease intervention. EVs are expected to become early diagnostic biomarkers of hypertension-induced chronic kidney disease [118]. Urine is an ideal specimen for detecting renal injury. In addition to the advantage of noninvasiveness, the EV-derived proteins which are contained in urine could also reflect the damage of renal cells [119]. Moreover, the level of PTC-EMPs (peritubular capillary endothelial microparticles), which are urinary exosomes positive for the peritubular capillary marker plasmalemmal-vesicle-associated protein, may be early biomarkers of renal injury independent of proteinuria in patients with hypertension [53]. The cyclin-dependent kinase (Cdk) inhibitor, p16^Ink4a^ (p16), is an ideal biomarker of cellular senescence [120]. The elevated level of p16^+^ EVs in the urine of patients with hypertension could reflect the increased proximal tubular cellular senescence [54]. In addition to the changes of EVs' own level, the miRNA contained in EV is also helpful to the diagnosis of hypertension [121]. The downregulated expression level of miR-192-5p and miR-204-5p from urinary exosomes would be helpful to diagnose patients with “nonclassical” apparent mineralocorticoid excess [55]. Early recognition of this phenotype helps to prevent the progression of arterial hypertension. These examples demonstrate the unique diagnostic potential of EVs in hypertensive chronic kidney disease (Table 1).

#### 4.3.3. HF

Heart failure (HF) is a kind of myocardial systolic dysfunction caused by multiple factors, and it is also the last stage of various CVDs [97, 122]. Similar to other aging-related diseases, oxidative stress plays an important pathological role in CVDs. Exosomal miRNAs play pathogenic roles in HF by participating in oxidative stress [123, 124]. Nrf2 is considered as an amplifier of the antioxidant pathway [125], while miR-27a, miR-28-3p, and miR-34a contained in exosomes could mediate Nrf2 imbalance thereby promoting the development of HF [124].

As to the treatment of HF, EVs are favorable agents. Nakamura et al. [99] found that intravenous injection of human BMSCs could play a therapeutic role in mice with HF through EVs. Moreover, adiponectin can stimulate EV biogenesis and secretion by binding to T-cadherin on human BMSCs, thereby enhancing the curative effect. This provides a new strategy for solving the problem of EVs' production. Compared with other cell sources, cardiogenic EVs may have more therapeutic advantages [100, 126]. Studies have shown that exosomes derived from cardiac fibroblast-iPSCs have a better effect than those from dermal fibroblast-iPSCs in reducing cardiac remodeling [126]. Although the specific therapeutic mechanism of EVs remains unclear, it may be associated with the miRNAs in EVs [101]. Future studies should focus on elucidating the underlying molecular mechanisms (Table 2). At present, the evidence of EVs for HF diagnosis is not sufficient. Oh et al. [127] predicted miRNAs from EVs that may be biomarkers for HF diagnosis by comparing the EV miRNA expression profiles between normal mouse hearts and HF mouse hearts. However, further verification is still needed.

### 4.4. Roles of EVs in DM and Its Complications

DM is an aging-related metabolic disorder marked by a chronic elevation of blood glucose levels caused by insufficient insulin secretion or function defects [128]. At present, the prevalence of type 2 DM (T2DM) is the highest, followed by type 1 DM (T1DM), while other types of DM account for a small proportion [128]. Chronic hyperglycemia in DM causes damage to blood vessels, which can lead to a series of DM-associated complications [129]. Diabetes is considered as an inducement to accelerate cellular senescence, and it is associated with aging-related cardiovascular diseases and kidney diseases caused by hyperglycemia [130]. This highlights the link between aging-related diseases. DM has become a global health problem in recent years due to aging populations, which makes it essential to identify effective molecular markers and drug targets for DM.

#### 4.4.1. T2DM

The onset of T2DM usually occurs after the age of 40, and it is considered to be a typical aging-related disease [131]. With the development of T2DM and its cardiovascular complications, EVs change both in quantity and quality [132]. By analyzing EVs isolated from patients' plasma, Masi et al. [56] reported an EV biomarker combination containing five differentially expressed miRNAs (miR-141-3p, miR-324-5p, miR-376c-3p, miR-26b-5p, and miR-374b-5p) and three proteins (immunoglobulin heavy constant gamma 1, interalpha-trypsin inhibitor, and heavy chain H2 and serotransferrin), which had a good indication effect on the prognosis of DM complications. Aside from being biomarkers, EVs can also be used as therapeutic targets for DM. T2DM is characterized by insulin resistance, and Kumar et al. [133] reported that high-fat diet-induced exosomes might contribute to insulin resistance. As a result, intestinal exosomes can serve as a wide range of therapeutic targets. In addition, EVs from other sources may be available for T2DM treatment [102, 103, 134] (Table 2).

#### 4.4.2. Diabetic Foot Ulcer

There is no doubt that diabetic foot ulcer is a serious complication of DM that negatively impacts patients' quality of life. In recent years, increasing evidence has pointed that MSC-EVs could be a potentially effective agent for diabetic wounds [135]. For example, Pomatto et al. [136] found that BMSC-EVs primarily promoted cell proliferation, while ADSC-derived EVs (ADSC-EVs) showed significant ability to promote endothelial cell migration and angiogenesis, which may be related to their expression of specific molecules. Notably, studies have shown that pretreatment of MSCs with chemical or biological factors could enhance the biological activity of MSC-Exos. For example, BMSC-Exos pretreated with atorvastatin (ATV) had better effects than nonpretreated BMSC-Exos both *in vivo* and *in vitro* [137]. Furthermore, the combination of pluronic F-127 (PF-127) hydrogel and hucMSC-derived exosomes could significantly enhance wound healing and promote granulation tissue regeneration [138]. PF-127 thermosensitive hydrogels could carry and sustainably release exosomes, so biomaterial-based exosome therapy may be helpful for diabetic wound healing. In addition to MSC-EVs, circulating exosomes isolated from patients with DM may also be used for treating diabetic foot ulcers [139, 140]. Taken together, the available evidence encourages further studies to explore the potential of EVs as a future diagnostic and therapeutic tool for diabetic foot ulcer.

#### 4.4.3. Diabetic Nephropathy

Diabetic nephropathy (DN) is one of the microvascular complications of DM, which causes end-stage renal disease [141]. Its clinical diagnosis mainly depends on the presence of proteinuria and the estimated decrease in the glomerular filtration rate [142]. However, renal function may deteriorate before microalbuminuria can be detected [143]. Therefore, more sensitive biomarkers are required for DN diagnosis. According to recent studies, urinary EVs might be potential noninvasive biomarkers for early diagnosis and treatment of DN [57, 144].

Currently, the treatment of DN is divided into two main areas: (i) early treatments that include strict control of blood sugar and blood pressure to prevent DN from developing and (ii) comprehensive treatments for advanced DN that include dialysis or kidney transplantation [145]. However, the incidence of end-stage renal disease remains high. BMSCs-Exos have been proven to participate in slowing down the progression of DN by controlling hyperglycemia and protecting kidney function [141]. In addition, exosomes derived from ADSCs and hucMSCs have also been confirmed to be used for the treatment of DN [146, 147] (Table 2). These studies have laid the foundation for the application of EVs as a new biological therapy for DN. However, the protective mechanism of EVs on DN requires further researches.

#### 4.4.4. Diabetic Retinopathy

The early stages of diabetic retinopathy (DR) do not cause any symptoms, but if left unchecked, it can cause significant retinal damage [148]. Recently, researchers have found that miR-431-5p in serum-derived EVs is upregulated in proliferative diabetic retinopathy (PDR) patients [58]. In addition, two other studies also reported that miR-150-5p, miR-21-3p, and miR-30b-5p extracted from circulating EVs may serve as biomarkers for predicting DR [59, 60]. Except for miRNAs, it is indicated that TNFAIP8 was upregulated in both plasma small extracellular vesicle and vitreous of DR patients [61]. The collection of these molecules will be helpful to DR diagnosis. In the treatment of DR, miR-192 in MSC-EVs could target and negatively regulate ITGA1, thereby ameliorating diabetic retinal damage by decreasing the inflammatory response and angiogenesis [149]. Similarly, hucMSC-derived small EVs could upregulate miR-18b and reduce retinal vascular leakage and retinal thickness [150]. Overall, these findings provide new insights into EV-based therapy for DR.

#### 4.4.5. Diabetic Macrovascular Complications

Macrovascular complications of DM include accelerated cardiovascular disease, which causes myocardial infarction, and cerebrovascular disease, which manifests as stroke. It has been reported that EVs could be used to treat diabetic macrovascular diseases. For example, Venkat et al. [151] reported that CD133^+^ exosomes upregulated miR-126 expression and reduced the expression of myocardial inflammatory factors, thus improving cardiac function of T2DM stroke mice. Other studies have also reported favorable therapeutic effects of EVs [12, 152]. Liu et al. [153] proved that increased levels of miR-1443p in diabetic exosomes could weaken endothelial progenitor cells' ability to mobilize. It may be possible to improve cardiac repair after myocardial infarction by using enriched miR-1443p.

### 4.5. Roles of EVs in Skin Aging

Human skin is a finely structured organ that acts as a natural shield, sensor, and alarm of the body [154]. Both internal and external factors are strong incentives for skin changes. As the main external cause of skin aging, ultraviolet (UV) has strong skin penetration ability and induces skin photoaging [155]. Although there are differences in the clinical features and histological characteristics in intrinsic and extrinsic skin aging [156], the underlying molecular pathways are similar: extracellular matrix (ECM) degradation caused by MMP overexpression [157]. Furthermore, aging skin shows a higher proportion of senescent cells, and aging microenvironment constructed by gradually accumulated senescent cells is easier to accelerate skin aging [32].

Stem cells can theoretically solve the problem of collagen loss in aging skin. At present, stem cells for injection mainly come from autologous adipose tissue [158], but this method is expensive and risky, thereby limiting its prevalence. Besides, the clinical safety of iPSC therapy remains uncertain due to the introduction of oncogenes. Skin antiaging goes through a complex process of skin tissue repair and skin function recovery. Under this complexity, efficient communication between skin cells is essential. EV-mediated cell information exchange is widely involved in the regulation of skin cell function [159]. In recent years, their strong roles in the proliferation of epidermal cells and the recovery of dermal cells' vitality made them potential drugs to reverse skin aging. Here, we explored the different effects of several EVs against skin aging.

UV can directly contribute to the decline of human dermal fibroblast (HDF) function. Choi et al. [160] observed that human ADSC-EVs could alleviate the damage of HDF migration and proliferation ability caused by UVB irradiation. Further study revealed that EV treatment could upregulate the level of tissue inhibitors of MMP-1 and TGF-*β*1 in UV-irradiated HDF cells and then inhibit the degradation of collagen. In addition, the increase of ROS induced by UV has a major influence in photoaging [157]. On the one hand, ROS may be a necessary signal messenger for melanin production, which protects against UVA-induced skin reaction [161]. However, on the other hand, excessive ROS will lead to DNA damage, inflammatory reactions, decreased production of antioxidants, and increased MMP expression in skin cells. Our past study have shown that hucMSC-Exos rich in 14-3-3*ζ* could upregulate the expression of SIRT1 in skin keratinocytes, thereby inhibiting oxidative stress and autophagy activation induced by UV irradiation [162]. Besides, exosomes derived from HDF could reduce skin wrinkles in nude mice caused by UVB irradiation, and some SASP factors were also relatively reduced [163]. Aging skin appears as functional deterioration and shows an increased proportion of senescent skin cells [164, 165]. The immune homeostasis function of macrophages is impaired with age, resulting in the decline of its selective scavenging ability to aging cells. This will contribute to the abnormal accumulation of senescent cells in skin [166]. However, there is little research on how UV-induced senescent cells bypass immune clearance. An effective skin rejuvenation strategy may involve applying EVs to restore the immune surveillance ability from aging skin. It may be feasible to externally supplement EVs from young macrophages to promote the recovery of the function of aging macrophages. And it may be an important research direction to analyze the differences between homogeneous EVs from young and aging macrophages to find possible beneficial molecules. Hence, further research is required to elucidate how to delay skin aging by regulating the immune activity of macrophages through EVs. Because of the existence of the skin barrier, simply applying EVs to the skin surface will sharply reduce its effectiveness. Studies have shown that ADSC-EVs combined with a microneedle roller can effectively reduce the aging phenotype of SKH-1 mice [167], but this method of promoting EV absorption could easily increase skin sensitivity. And in recent years, the microneedle patch has become a research hotspot in the field of dermatology based on its advantages of minimal invasiveness, painlessness, and high drug loading. However, this transdermal drug delivery system requires special equipment and faces the risk of failure of preloaded active substances. Thus, modifying the physical properties of EVs while maintaining its activity has become a challenge for the exogenous supplement of EVs in the field of skin antiaging.

## 5. Conclusions and Perspectives

Cellular senescence and aging are inseparable. Although some mechanisms leading to cellular senescence and many antiaging targets have been found, this may only be the tip of the iceberg of aging. Further clarifying the aging mechanism is still the basis of antiaging treatment. EVs, especially exosomes, have been proven to participate in the regulation of various diseases and have shown their great potential in becoming biomarkers and therapeutic agents in aging-related diseases. Some studies on EVs have entered the stage of clinical trials, but challenges continue to exist when meeting clinical requirements. First, the current research of EVs mainly focused on whether they have curative effects, but which component of EVs take effect is not comprehensive. This unknown factor raises doubts about the safety and effectiveness of EVs. Second, there is still a lack of strict standard in EVs' quality management. Different tissue sources, donor cells, and preparation methods will produce heterogeneous EVs, and with the inconsistency of the *in vivo* and *in vitro* models between laboratories, the effective concentration and intervention methods of EVs in different diseases have not been finalized, which hinders their clinical transformation. Moreover, EVs are natural drug carriers, and the appropriate ratio to drugs is the important premise for their function; therefore, a scientific matching system is needed. Besides, regarding the problem of low EV yield and purification efficiency, some researchers found that human iPSC could produce EVs several times higher than MSC under specific culture conditions, and these iPSC-EVs could be efficiently ingested by target cells [168]. This suggests that human iPSC as the source cell of EVs may become a more promising choice in the field of antiaging. Finally, the role of standalone therapy is always limited. Exploring the combined medication of EVs and other effective drugs may become the trend of development in the future.

Despite the challenges, beneficial achievements have been made in the field of EVs in recent years. With the continuous maturity in separation, purification, and identification standards, EVs are expected to be candidates for the diagnosis and treatment of clinical aging-related diseases. Moreover, preventing aging is an urgent need of developed society, and the research on the preventive efficacy of EVs in aging-related diseases may become a new research direction of modern medicine.

## Figures and Tables

**Figure 1:** Biogenesis, secretion, and uptake of exosomes. Exosome is a subset of EVs. The biogenesis of exosomes mainly goes through the stages of endocytosis and MVB formation. Different nucleic acids or proteins are loaded during the formation of exosomes. These cargoes can be internalized into recipient cells through different mechanisms, thus realizing the information transmission function of exosomes. Moreover, some cargo proteins can also be used as biomarkers for the identification of exosomes.

**Figure 2:** The stimuli and identification of cellular senescence. Cellular senescence has two sides. On the one hand, cellular senescence can promote tissue remodeling and inhibit tumor development. On the other hand, accumulation of senescent cells can lead to a variety of aging-related diseases. Cellular senescence is caused by different stimuli, and the mechanism of cellular senescence is very complex. Therefore, the identification of senescent cells needs to be analyzed from different aspects.

**Figure 3:** The roles of EVs in aging-related diseases. EVs derived from normal cells have therapeutic effects on aging-related diseases. There are many sources of natural EVs, and the optimal selection should consider the yield, targeting, and curative effect. In addition, EVs are also high-quality drug delivery systems (DDSs), which can target the delivery of therapeutic drugs through engineered EVs. EVs derived from senescent cells will contribute to the transmission of aging information and further promote the accumulation of senescent cells, which may eventually lead to aging-related diseases. Significantly, EVs derived from these senescent cells are also potential diagnostic biomarkers and therapeutic targets.

**Table 1:** EVs and their cargoes as biomarkers of aging-related diseases.

Disease	Nanovesicle	Source of EVs	Biomarkers	Refs.
AD	NDEs	Human blood	GAP43, neurogranin, SNAP25 and synaptophysin 1↓	[34]
	Exosomes	Human serum	Gelsolin↓	[40]
	NDEVs	Human plasma	A*β*42, p181-tau, and MMP-9↑	[41]
	EVs	Human plasma	The size of EVs↑ The number of EVs↓	[42]
	NEVs	Mouse plasma	t-tau, p181-tau, and A*β*42↑	[43]
	NEVs	Human serum	p181-tau, p231-tau, and annual rate of change in insulin signaling biomarkers↑	[39, 44]
	NDEs	Human plasma	A*β*1-42↑ SS-16 scores↓	[45]
Hypertension	Exosomes	Urine	PTC-EMPs↑	[53]
	EVs	Urine	p16^+^ EVs↑	[54]
	Exosomes	Urine	miR-192-5p and miR-204-5p↓	[55]
T2DM	EVs	Human plasma	IGHG-1, miR-324-5p, miR-376c-3p, and miR-374b-5p↓ ITIH2 protein, serum ferritin, miR-141-3p, and miR-26b-5p↑	[56]
DN	Exosomes	Urine	miR-4534↑	[57]
DR	EVs	Human serum	miR-431-5p↑	[58]
	EVs	Human plasma	miR-150-5p↓ miR-21-3p, and miR-30b-5p↑	[59, 60]
	Small EVs	Human plasma	TNFAIP8↑	[61]

Abbreviations: NEVs: neuronal extracellular vesicles; NDEVs: neuronally derived extracellular vesicles; NDEs: neuronal-derived exosomes; IGHG-1: immunoglobulin heavy constant gamma 1; ITIH2 protein: interalpha-trypsin inhibitor heavy chain H2 protein; TNFAIP8: tumor necrosis factor-*α*-induced protein 8.

**Table 2:** Therapeutic effects of EVs from different sources in aging-related diseases.

Disease	Source of EVs	Animal model	Mechanism(s) and effect(s)	Refs.
AD	NSCs	APP/PS1 mice	Increased the metabolism and function of mitochondria, the activation of SIRT1, and the activity and integrity of synapses; decreased the oxidative damage of cerebral cortex and the inflammatory response	[46]
	hNSCs	5xFAD mice	Mitigated AD-related behavioral and molecular neuropathologies	[47]
	MSCs	J20 AD transgenic (Tg) mice	Improved brain metabolism and cognitive function; reduced A*β* plaque load and inhibited astrocyte activation	[48]
	MSCs	3xTg AD mice	Dampened microglia activation and reduced dendritic spine loss	[49]
	ADMSCs	APP/PS1 mice	Decreased the release of inflammatory factors by inhibiting pyroptosis	[50]
	HAs	APP/PS1 mice	HA-Exo provided neuroprotective effects to reverse oligomeric amyloid-*β*-induced cytotoxicity *in vitro*	[51]
	Mouse plasma	OA-induced AD mice	Reduced the formation of insoluble NFTs and inhibited CDK5-mediated phosphorylation of tau	[52]

Osteoporosis	BMSCs	OVX-induced postmenopausal osteoporosis mice	miR-29b-3p in EVs potentiated osteogenic differentiation through SOCS1/NF-*κ*B pathway	[63]
	Serum of young rats	OVX-induced postmenopausal osteoporosis mice	miR-19b-3p in EVs promoted the osteogenic differentiation of BMSCs	[78]
	hucMSCs	OVX-induced postmenopausal osteoporosis mice and TS-induced hindlimb disuse osteoporosis mice	CLEC11A in EVs promoted the shift from adipogenic to osteogenic differentiation of BMSCs and inhibited bone resorption	[81]
	BMSCs	OVX-induced postmenopausal osteoporosis mice	MALAT1 in EVs promoted osteoblast activity through microRNA-34c/SATB2 axis	[82]
	SHED	OVX-induced postmenopausal osteoporosis mice	miR-346 in EVs rescued impaired BMSC function and recovered bone loss	[83]
	Mid-to-late stage of osteoblasts	OVX-induced postmenopausal osteoporosis mice	Enhanced osteogenesis	[84]
	BMSCs	OVX-induced postmenopausal osteoporosis mice	miR-150-3p in EVs promoted osteoblast proliferation and differentiation	[85]
	BMSCs	OVX-induced postmenopausal osteoporosis mice	miR-29a in EVs promoted angiogenesis and osteogenesis by acting on human venous endothelial cells	[86]
	BMSCs	OVX-induced postmenopausal osteoporosis mice	miR-22-3p in EVs promoted osteogenic differentiation through MYC/PI3K/AKT pathway	[87]
	ECs	OVX-induced postmenopausal osteoporosis mice	miR-155 in EVs inhibited osteoclasts activity by acting on BMMs	[88]
	Bovine milk	OVX-induced postmenopausal osteoporosis mice	Reduced osteoclast presence through RANKL/OPG system	[90]
	Bovine colostrum	GIOP mice	Facilitated preosteoblast proliferation and inhibited osteoclast differentiation	[91]
	hAFSCs	GIOP mice	Ameliorated the differentiation ability of HOB through a redox-dependent regulation of SIRT1	[92]
	hUCB	OVX-induced postmenopausal osteoporosis mice	miR-3960 in EVs promoted osteogenesis and inhibited osteoclastogenesis	[93]

Hypertension	Plasma from WKY	SHR and WKY	Modulated systemic blood pressure as well as structure and function of cardiovascular tissues in both normotensive and hypertensive rats	[94]
	CDCs	Ang II-induced male C57BL/6J mice	EV-YF1 attenuated cardiac hypertrophy and renal injury induced by Ang II infusion, without affecting blood pressure	[95]
	iPS-MSCs	Young and old male C57BL/6 mice	Attenuated aging-associated vascular endothelial dysfunction, arterial stiffness, and hypertension through SIRT1-AMPK*α*-eNOS pathway	[96]
	Vascular adventitial fibroblasts of normal rats	SHR and WKY	miR-155-5p in EVs inhibited cell migration and proliferation in VSMCs of SHR through suppressing ACE expression, oxidative stress, and inflammation	[97, 98]

HF	hBMSCs	TAC-operated C57B6/J male mice	Regulated the fibrogenic and adhesion pathways, and cellular metabolic process in the damaged heart	[99]
	Normal human cardiomyocytes	Diseased heart tissues received from patients who underwent heart transplantation at UNC Hospital after heart failure	Promoted cardiomyocyte proliferation, decreased programmed cell death, and stimulated angiogenesis *in vitro* through phosphatase and tensin homolog/Akt pathway	[100]
	iPSC-Pg and iPSC-CMs	Nude mice with permanent left anterior coronary artery occlusion	miRNAs in EVs are effective in the treatment of CHF	[101]

T2DM	hucMSCs	Low concentrations of TNF-*α* and high glucose medium were used to simulate insulin resistance in human adipocytes	The insulin-stimulated glucose uptake↑ The level of leptin↓ The mRNA expression of sirtuin-1 and insulin receptor substrate-1↑	[102]
	Pancreatic *β* cells	*β* cell-specific miR-29a/b/c transgenic mouse (*β*TG) model	Prediabetic *β* cells release exosomal miR-29 to reset macrophage inflammatory tone	[103]

Abbreviations: hNSCs: human neural stem cells; ADMSCs: adipose-derived mesenchymal stem cells; OA: okadaic acid; CDK-5: cyclin-dependent kinase 5; OVX-induced: ovariectomized-induced; GIOP: glucocorticoid-induced osteoporosis; SHED: stem cells from human exfoliated decimal teeth; BMMs: bone marrow-derived macrophages; TS-induced: tail suspension-induced; SHR: spontaneous hypertensive rat; WKY: Wistar-Kyoto rat; iPS-MSCs: induced pluripotent stem cell-derived mesenchymal stem cells; SIRT1-AMPK*α*-eNOS: sirtuin type 1-AMP-activated protein kinase alpha-endothelial nitric oxide synthase; ACE: angiotensin-converting enzyme; CDCs: cardiosphere-derived cells; Ang II: angiotensin II; TAC: transverse aortic constriction; iPSC-Pg: human induced pluripotent stem cell-derived cardiovascular progenitor; iPSC-CM: human induced pluripotent stem cell-derived cardiomyocyte; CHF: chronic heart failure.
